# Thyroid Nodule Classification in Ultrasound Images by Fusion of Conventional Features and Res-GAN Deep Features

**DOI:** 10.1155/2021/9917538

**Published:** 2021-07-22

**Authors:** Yuan Hang

**Affiliations:** School of Electronic Information and Electrical Engineering, Shanghai Jiao Tong University, Shanghai, China

## Abstract

In spite of the gargantuan number of patients affected by the thyroid nodule, the detection at an early stage is still a challenging task. Thyroid ultrasonography (US) is a noninvasive, inexpensive procedure widely used to detect and evaluate the thyroid nodules. The ultrasonography method for image classification is a computer-aided diagnostic technology based on image features. In this paper, we illustrate a method which involves the combination of the deep features with the conventional features together to form a hybrid feature space. Several image enhancement techniques, such as histogram equalization, Laplacian operator, logarithm transform, and Gamma correction, are undertaken to improve the quality and characteristics of the image before feature extraction. Among these methods, applying histogram equalization not only improves the brightness and contrast of the image but also achieves the highest classification accuracy at 69.8%. We extract features such as histograms of oriented gradients, local binary pattern, SIFT, and SURF and combine them with deep features of residual generative adversarial network. We compare the ResNet18, a residual convolutional neural network with 18 layers, with the Res-GAN, a residual generative adversarial network. The experimental result shows that Res-GAN outperforms the former model. Besides, we fuse SURF with deep features with a random forest model as a classifier, which achieves 95% accuracy.

## 1. Introduction

Thyroid nodules refer to solid or fluid-filled lumps in the thyroid, radiologically distinct from surrounding parenchyma [1]. Although most of them are not serious, there are still a small percentage of thyroid nodules which are cancerous. Thyroid nodules are prevalent, especially among women and older populations. In the United States, the estimated annual incidence of thyroid nodules is approximately one per thousand per year.

Thyroid ultrasonography (US) is a noninvasive, inexpensive procedure widely used to detect and evaluate the thyroid nodules. It plays an important role in providing information such as the nodule positions, dimensions, structure, and thyroid pathologic changes [2]. Thyroid US has been confirmed to be an effective way to distinguish benign lesions from malignant ones. Several US features, such as taller than wider shape, blurred margins, hypoechogenicity, microcalcification, and solid appearance, have been found to be suggestive of malignant lesions, while US findings such as hyperechogenicity, coarse calcification, and cystic appearance are highly suggestive of benign ones.

The ultrasonography method for image classification is a computer-aided diagnostic (CAD) technology based on image features. Under the help of deep learning and cloud technology, the establishment of an intelligent diagnosis model based on image classification can provide an accurate, stable, highly efficient, and reproducible ultrasound diagnosis pathway for thyroid nodules, which can effectively reduce workload and diagnostic differences among physicians.

In 1943, McCulloch and Pitts established a simple neural network model with electrical circuits, which indicates the first step toward artificial neural networks [3]. Then in 1998, LeCun proposed a simple convolution neural network (CNN) named LeNet-5 for handwritten character recognition and promoted the development of deep learning [4]. A simple CNN is a collection of sequential layers, including convolutional layer, max-pooling layer, and fully connected layer. The convolutional layer is the most substantial block of a CNN, which does most of the heavy computing work, while the max-pooling layer between convolutional layers is designed to reduce the scale of parameters and computation in the network, including some noise. The fully connected layer plays a classifier's role in the convolutional neural network. In 2012, AlexNet, a GPU implementation of CNN, marked a breakthrough in deep learning [5]. On one hand, AlexNet introduces Rectified Linear Unit (ReLU) activations instead of sigmoid, tanh, and SoftMax to vanishing gradients. On the other hand, it uses a regularization technique called dropout to reduce overfitting. Goodfellow and his fellows proposed the GAN in 2014, to generate models through adversarial process [6]. It is an unsupervised learning task composed of two submodels, a discriminator and a generator. The generator part learns from the data distribution and creates fake data. The discriminator part then tries to estimate the probability and distinguish the real data from the fake ones transmitted from the generator. Most GANs nowadays are based on the Deep Convolutional Generative Adversarial Networks (DCGANs) architecture [7].

Biomedical imaging is composed of X-ray, CT, MRI, PET, US, and so on. Kawahara focused on the classification task for skin lesions. He proposed multiresolution-tract CNN architecture in [8]. Each tract from various resolutions has the chance to learn interactions across multiple resolutions. It lies on the mechanism that all of these tracts share the same field-of-view. Jiao has undertaken some research on breast mass classification tasks in [9]. The network combines both the intensity information and the deep features to predict the ground truth of test images and simulate the diagnostic procedure. In [10], Tajbakhsh intends to detect and distinguish lung nodules with a comparison between MTANNs and CNNs.

As part of our work, we illustrate an end-to-end method which involves the combination of the deep features with the conventional features together to form a hybrid feature space. End-to-end methods make it possible to directly map the raw input to the desired output and eliminate the need for hand-crafted features. The conventional features we use in this paper contain HOG, LBP, SIFT, and SURF. Before feature extraction, we explore several existing image enhancement techniques, such as histogram equalization, Laplacian operator, logarithm transform, and Gamma correction, to enhance the quality and characteristics of origin input we access. Several preliminary experiments are conducted to have a comparison on the accuracy of various image enhancement techniques and feature extraction solutions. Finally, we combine them with deep features of residual generative adversarial network. We compare the ResNet18, a residual convolutional neural network with 18 layers, with the Res-GAN, a residual generative adversarial network. The experimental result shows that Res-GAN outperforms the former model. Besides, we fuse SURF with deep features with a random forest model as a classifier, which achieves 95% accuracy.

The paper is structured in detail as follows.  Section 2 presents some essential information about the dataset we use in our experiment and the theoretical basis of image classification process, which can be further divided into several subprocesses, such as image enhancement, feature extraction, and classifiers.  Section 3 presents the corresponding experimental results for the methodology.  Section 4 gives a conclusion for our efforts.

## 2. Methodology

### 2.1. Dataset

The data come from an open-source thyroid nodule image dataset named TDID [11]. It contains US nodular thyroid images from nearly three hundred patient cases from various ages, genders, and different ultrasound machine sources.

As shown in Table 1, we choose one or several US images for each patient. There are 428 samples in total, around 60% for training set and around 40% for testing set. We use 5-fold cross-validation in our experiment to avoid overfitting.

Each ultrasound image is provided with its ground truth class (benign or malignant) by expert radiologists. We list some typical cases here. US findings such as round shape, smooth margin, coarse calcification, hyperechogenicity, cystic appearance, and clear boundary are highly suggestive of benignity, as shown in Figure 1. On the contrary, several US features, such as taller than wider shape, blurred margins, microcalcification, hypoechogenicity, solid appearance, and unclear boundary, have been found to be indicative of malignant potential, as shown in Figure 2.

### 2.2. Image Enhancement

The US images are collected from different ultrasound machines, leading to imbalance in exposure. Before undertaking feature engineering, we are supposed to preprocess origin images, including noise reduction and image enhancement. Image enhancement is used to highlight certain information of some parts of an image. We introduce several commonly used image enhancement techniques for our experiment, which are histogram equalization, Laplacian operator, logarithm transform, and Gamma correction. Among these techniques, Laplacian operator is often applied for edge detection and the others for image contrast improvement.

Several preliminary experiments are conducted.

#### 2.2.1. Histogram Equalization

The histogram for an image represents the PDF value of the pixel values in the image over the entire gray scale range. If most of the pixels are concentrated in the low gray area, the image will appear dark, but if they are concentrated in the high gray area, it will appear bright.

Histogram equalization is to adjust the gray scale distribution of the image to make the distribution on the gray scale of 0∼255 more balanced. It is used to elevate the contrast of the image, thus improving the visual effect of the image. Histogram equalization is often applied on images with lower contrast to enhance their subtle details.

#### 2.2.2. Laplacian Operator

Laplacian operator is a second-order spatial derivative mask. It is often applied to an image for edge detection. The edge of an image is divided into two categories. One is the outward edge, and the other one is inward edge.

Operator to detect outward edge is called positive Laplacian operator. The center element of the mask should be negative, while the rest of the elements should be nonnegative. On the contrary, as for the inward edge, negative operator is applied.

#### 2.2.3. Logarithm Transform

Logarithm transform can expand the gray value of parts of the image with gray values near zero to show more details. On the contrary, the part with higher gray value will be compressed and convey less information. Transformation method can be expressed as

(1) $$\begin{array}{c} \tilde{H}\left(x,y\right)=255\times \frac{\log\left(H\left(x,y\right)+1\right)-\min\left\{\log\left(H\left(x,y\right)+1\right)\right\}}{\max\left\{\log\left(H\left(x,y\right)+1\right)\right\}-\min\left\{\log\left(H\left(x,y\right)+1\right)\right\}}. \end{array}$$

#### 2.2.4. Gamma Correction

Gamma correction is mainly used to correct pictures with biased gray scale and also enhance their contrasts. It works well when the image contrast is low and the brightness is high. It depends on the value of *γ*. In case *γ* > 1, it is similar to logarithm transform.

Transformation method can be expressed as

(2) $$\begin{array}{c} \tilde{H}\left(x,y\right)=255\times {\left(\frac{H\left(x,y\right)}{\max\left\{H\left(x,y\right)\right\}}\right)}^{1/\gamma }. \end{array}$$

### 2.3. Feature Extraction

Feature extraction is crucial for multimedia processing. It is a part of the dimensionality reduction process. The conventional features are fused with deep features to form a hybrid feature space. We introduce several commonly used feature extraction methods for our experiment, which are HOG, LBP, SIFT, and SURF. Liu raised up a feature extraction methodology based on CNNs to combine HOG and SIFT together as part of the hybrid feature space [12].

Several preliminary experiments are conducted.

#### 2.3.1. Histogram of Oriented Gradient

HOG is an effective tool for object recognition. It is used to extract information related to pixel colors. The steps of HOG include

- current_cell ← current_size
- current_position ← cell_*i*_
- for *i* ∈ current_cell do
- histogram_*i*_ ← gradient_within_cell
- gradient ← Normalization
- end for
- HOG⟵histogram_in_each_cell

#### 2.3.2. Local Binary Pattern

The local binary pattern vector is obtained by comparing the gray value of the target pixel with the gray value of neighboring pixels. The specific process can be divided into three steps.

#### 2.3.3. Speed Up Robust Feature

SIFT is confirmed to be a mature method to detect the key points. However, it is comparatively slow. SURF, as an optimization of SIFT, speeds up the time efficiency and makes it more practical. Different from SIFT, SURF makes use of the Hessian matrix determinant approximation images to construct a pyramid scale space, as shown in Figure 3.

### 2.4. Classifier

#### 2.4.1. Residual Generative Adversarial Network

GAN is an unsupervised learning task composed of two submodels, a discriminator and a generator, as shown in Figure 4. The generator part analyzes the data distribution and creates fake data. The discriminator part learns to estimate the probability and distinguish the real data from the fake ones transmitted from the generator. Most GANs nowadays are based on the Deep Convolutional Generative Adversarial Networks (DCGANs) architecture. In Res-GAN, the generator is coupled with a deep residual network. The reason why we choose residual network here is that the residual mapping can learn the identity function more easily.

The generated picture and the real picture are, respectively, added with Gaussian noise and then input into the discriminator. The discriminator we establish for our Res-GAN is composed of one convolutional layer, one max-pooling layer, six residual modules, one average-pooling layer, and a fully connected layer successively. The input image first passes through a convolutional layer with a core size of 7 × 7 and a channel number of 64 and then enters the residual network structure after batch normalization. The residual network structure is composed of six residual network modules. The size of the convolution kernel of each module is 3 × 3, and the number of channels is 64, 64, 128, 128, 256, and 512, respectively. The input layer of the two fully connected layers is composed of the output features of the residual modules with different numbers of channels, and each module is spliced together, with a total of 960 dimensions.

The first fully connected layer (authenticity judgment layer) is used to judge whether the picture is a real picture or a generated picture. The authenticity judgment layer outputs a value through the Sigmoid activation function. When the value is greater than 0.5, it is judged as a real picture; otherwise, it is regarded as a generated picture.

The second fully connected layer (good and evil judgment layer) is used to judge whether the picture is benign or evil. The good and evil judgment layer outputs a two-dimensional vector through the SoftMax activation function, and the column corresponding to the larger value in the vector is the label category. Among them, 1 means malignant and 0 means benign. The real picture comes with its own benign and malignant label, and the benign and malignant label of the generated picture is the label of the input generator.

## 3. Evaluation

### 3.1. Metrics

Through the classifier, the outcomes can be divided into four groups, which are TP, TN, FP, and FN. TP stands for the proportion of malignant (positive) cases that are correctly classified as malignant ones, while TN stands for the proportion of benign (negative) cases that are correctly classified as benign ones. FP stands for the proportion of benign (negative) cases that are incorrectly classified as malignant ones, while FN stands for the proportion of malignant (positive) cases that are incorrectly classified as benign ones. Based on these definitions, we use accuracy, specificity, and sensitivity as the metrics of our experiment.

(3) $$\begin{array}{c} \text{Accuracy}=\frac{\text{TP}+\text{TF}}{\text{TP}+\text{TF}+\text{FP}+\text{FN}},\\ \text{specificity}=\frac{\text{TN}}{\text{TN}+\text{FP}},\\ \text{sensitivity}=\frac{\text{TP}}{\text{TP}+\text{FN}}. \end{array}$$

### 3.2. Experiment for Image Enhancement

We introduce several image enhancement techniques. A preliminary experiment is designed to have a contrast of the effectiveness among these techniques. We apply each image enhancement technique on the noise-reduced images. Here, we use a traditional machine learning classification algorithm. We use HOG as the feature and use the random forest as the classifier. We evaluate the effectiveness in two aspects. One is the visual effect, which is shown in Figure 5. All methods increase the exposure of the image, while Laplacian operator and Gamma correction do mere work. The other one aspect is quantized. The metrics are shown in Table 2. We use 69.3% as our baseline. After applying the Logarithm transform, the accuracy drops a lot, while other methods merely increase the accuracy. Among these, histogram equalization outperforms the rest. From the subjective and objective aspects, we finally choose histogram equalization as our image enhancement method.

As for the image enhancement process, we have decided what technique we use. Besides, we also need to decide what target we apply. We have a contract on different data pairs. To simplify the problem, we still take HOG as our input feature and use the random forest as our classifier. The experiment result is shown in Table 3. One interesting finding is that when we apply image enhancement on the whole training dataset, the accuracy drops for about 5.4%, which is out of our expectations. As a result, we only apply histogram equalization on the malignant cases in the training set to improve classification effectiveness.

### 3.3. Experiment for Feature Extraction

We introduce several feature extraction techniques. A preliminary experiment is designed to have a contrast of the effectiveness among these techniques. We apply each image enhancement technique on the noise-reduced images. Among these methods, HOG and LBP are designed to detect the edge of the image as shown in Figures 6(a) and 6(b). The SIFT and SURF are designed to detect the key joint of the image. As shown in Figures 6(c) and 6(d), SURF outperforms SIFT. The quantized experimental result is shown in Table 4. As for each method, we adjust the parameters to achieve the best result. The accuracy ranges from 71% to 74%.

### 3.4. Experiment for Classifier

As our dataset is small, we rotate and slip the origin dataset to augment the scale of the dataset. We have a contrast of our Res-GAN model and ResNet18, which is a convolutional neural network with 18 layers. The experimental result is shown in Table 5. It is obvious that Res-GAN outperforms the ResNet18 model.

We combine the conventional feature and the deep feature as a hybrid feature space for a further classifier. We use SIFT and SURT as the feature candidate here. Besides, we have a contrast of two classifiers. One is the random forest and the other is AdaBoost. The experimental result is shown in Table 6. In the case that we combine deep features with SURF feature and use random forest as a classifier could we reach accuracy at 95%.

## 4. Conclusion

In this paper, we illustrate a method which involves the combination of the deep features with the conventional features together to form a hybrid feature space. Several image enhancement techniques, such as histogram equalization, Laplacian operator, logarithm transform, and Gamma correction, are undertaken to improve the quality and characteristics of image before feature extraction. Among these methods, applying histogram equalization not only improves the brightness and contrast of the image but also achieves the highest classification accuracy at 69.8%. We extract features such as HOG, LBP, SIFT, and SURF and combine them with deep features of residual generative adversarial network. We compare the ResNet18, a residual convolutional neural network with 18 layers, with the Res-GAN, a residual generative adversarial network. The experimental result shows that Res-GAN outperforms the former model. Besides, we fuse SURF with deep features with a random forest model as a classifier, which achieves 95% accuracy.

## Figures and Tables

**Figure 1:** Ultrasound image of benign cases. (a) Round shape; (b) smooth margin; (c) coarse calcification; (d) hyperechogenicity; (e) cystic appearance; (f) clear boundary.

**Figure 2:** Ultrasound image of malignant cases. (a) Taller than wider shape; (b) blurred margin; (c) macrocalcification; (d) hypoechogenicity; (e) solid appearance; (f) unclear boundary.

**Figure 3:** SURF approximation.

**Figure 4:** Res-GAN architecture.

**Figure 5:** Comparison of image enhancement technique. (a) Histogram equalization; (b) Laplacian operator; (c) logarithm transform; (d) Gamma correction.

**Figure 6:** Comparison of feature extraction methods. (a) HOG; (b) LBP; (c) SIFT; (d) SURF.

**Table 1:** Dataset distribution.

	Training set	Testing set	Total
Benign	43	38	71
Malignant	214	143	357
Total	257	171	428

**Table 2:** Comparison of image enhancement technique (%).

Group	Baseline	Histogram equalization	Laplacian operator	Logarithm transform	Gamma correction
Accuracy	69.3	69.8	69.6	67.0	69.6

**Table 3:** Comparison of image enhancement technique on different data targets (%).

Group	Baseline	Malignant only	Both benign and malignant
Accuracy	69.3	79.4	64

**Table 4:** Comparison of feature extraction technique (%).

Group	Parameter		Accuracy
HOG	Cell = (8, 8), block = (1, 1)		73.4
	Cell = (4, 4), block = (2, 2)		72.2
LBP	Radius = 2, *n* = 16		72.2
SIFT	Iter = 1	*k* = 100	68.5
		*k* = 1000	71.7
		*k* = 2000	71.1
		*k* = 3000	71.1
SURF	Iter = 1	*k* = 1000	71.9

**Table 5:** Comparison of ResNet18 and Res-GAN (%).

Group	Accuracy	Specificity	Sensitivity
ResNet18	82.2	66.2	89.8
Res-GAN	92.2	86.5	95

**Table 6:** Comparison of feature fusion by various classifiers (%).

	K-means iter	Random forest	AdaBoost
SIFT	1	93	92
	2	94	94
	3	93	93

SURF	1	95	93
	2	94	92

## Data Availability

The image data used to support the findings of this study have been deposited in the an open-access thyroid ultrasound image database repository (DOI: 10.1117/12.2073532).

## References

[1] Cooper D. S., Doherty G. M., Haugen B. R. (2009). Revised American thyroid association management guidelines for patients with thyroid nodules and differentiated thyroid cancer. *Thyroid*.

[2] Popoveniuc G., Jonklaas J. (2012). Thyroid nodules. *Medical Clinics of North America*.

[3] McCulloch W. S., Pitts W. (1943). A logical calculus of the ideas immanent in nervous activity. *Bulletin of Mathematical Biophysics*.

[4] LeCun Y., Bottou L., Bengio Y., Haffner P. (1998). Gradient-based learning applied to document recognition. *Proceedings of the IEEE*.

[5] Krizhevsky A., Sutskever I., Hinton G. E. (2012). Imagenet classification with deep convolutional neural networks. *Advances in Neural Information Processing Systems*.

[6] Goodfellow I. J., Pouget-Abadie J., Mirza M. (2014). Generative adversarial networks. https://arxiv.org/abs/1406.2661.

[7] Radford A., Metz L., Chintala S. (2015). Unsupervised representation learning with deep convolutional generative adversarial networks. https://arxiv.org/abs/1511.06434.

[8] Kawahara J., Hamarneh G. Multi-resolution-tract CNN with hybrid pretrained and skin-lesion trained layers.

[9] Jiao Z., Gao X., Wang Y., Li J. (2016). A deep feature based framework for breast masses classification. *Neurocomputing*.

[10] Tajbakhsh N., Suzuki K. (2017). Comparing two classes of end-to-end machine-learning models in lung nodule detection and classification: MTANNs vs. CNNs. *Pattern Recognition*.

[11] Pedraza L., Vargas C., Narváez F. An open access thyroid ultrasound image database.

[12] Liu T., Xie S., Zhang Y., Yu J., Niu L., Sun W. Feature selection and thyroid nodule classification using transfer learning.

